RETRACTED

# Signal Recognition Based on APSO-RBF Neural Network to Assist Athlete's Competitive Ability Evaluation

**DOI:** 10.1155/2021/4850020

**Published:** 2021-07-22

**Authors:** Feng Guo, Qingcheng Huang

**Affiliations:** Institute of Exercise Epidemiology and Department of Physical Education, Huaiyin Institute of Technology, Huai'an, Jiangsu 223003, China

## Abstract

The advanced analysis and research methods of big data will provide theoretical support for the integration of athletes' talent training. The advanced technological methods of big data will also give full play to the advantages of tapping the potential of talents and actively improve the success rate of grassroots young athletes. This paper proposes an improved Adaptive Particle Swarm Optimization (APSO) algorithm for the optimization of radial basis function (RBF) neural network parameters. The basic structure of RBF neural network is introduced, and the influence of parameters on the performance of RBF neural network is analyzed. The optimization method of RBF neural network parameters is analyzed, and Particle Swarm Optimization (PSO) algorithm is selected as the parameter optimization method of RBF neural network. In addition, an improved APSO algorithm is proposed according to the advantages and disadvantages of PSO and compared with other PSO algorithms. Experimental results show that the improved PSO algorithm has better accuracy. The improved PSO algorithm is applied to the parameter optimization of RBF neural network, and the experimental results prove the superiority of the proposed method. By weighting the second-level indicators, the weights of the second-level indicators of athletes' competitive ability are in order of skill, athletic quality, psychological ability, and artistic expression. Skills are the main factors that determine the level of competitive ability. Sports quality and psychological ability are important guarantees for supporting the normal performance of skills. Artistic expressiveness is a supplementary factor for competitive ability. The various elements cooperate with each other and interact with each other. The indicators do not exist alone but cooperate with each other to support the formation of the entire athletic ability system. In the content of the competitive ability index of excellent athletes, technical ability is the core, and sports quality, psychological ability, and artistic performance ability ultimately exist to serve the improvement of technical ability. The competition scores of the 100 athletes counted in this article are all above 9.0 points. The difference between APSO-RBF's action quality scores of 100 athletes and the real value is less than 3%. In terms of movement difficulty, the APSO-RBF evaluated athletes' scores are close to 1.65 points, which is basically the same as the real value.

RETRACTED

## 1. Introduction

In the current stage of athletes' grassroots training, the national competitive sports authorities have realized this problem and have begun to promote and advocate the thinking concept of objective data to guide athletes to grassroots coaches, especially in the training of national first- and second-level coaches [1]. The classroom teaching platform promotes the concept of applying big data to actual teaching and uses this method to try to solve the various ills caused by subjective judgments in the work of cultivating talents [2]. Therefore, objective data must be fully respected, and at the same time, the natural data of training continuously increases the amount of data and insists on using big data to monitor for a long time. On the other hand, from the perspective of athletes, it is also necessary to strengthen the thinking concept of taking objective data as the big one. To learn to be good at accumulating natural data, and at the same time expand the accumulated data on the time axis, you will find many problems that have not been paid attention to in the past [3].

An important feature of competitive sports is to continuously explore athletes' competitive potential to continuously improve their technical level. From the first Olympic Games to the present, the progress of sports training and the goals pursued by training are to best promote the improvement of athletes' physical level and maximize the development of athletes' competitive ability [4]. Competitive ability is the ability of athletes to effectively participate in training and competitions. It is composed of physical stamina, skills, mental abilities, and sports intelligence with different manifestations and different functions and is comprehensively manifested in the process of special training and competition [5]. Among them, the athlete's physical fitness refers to the basic athletic ability of the athlete's body, which is an important component of the athlete's competitive ability. Physical fitness is manifested through the athlete's morphological characteristics, the functions of various physiological systems, and athletic qualities. In the relationship between athletes' physical stamina, skills, and mental abilities, which are interrelated and restrict each other, physical stamina is the basis for forming athletes' skills, which is considerably larger than the hardware of athletic ability [6]. This characteristic determines that it is the material basis of competitive ability.

Radial Basis Function (RBF) neural network is a local approximation network. If the number of hidden layer nodes in the network is large enough, it can approximate any continuous function with arbitrary precision and has the global optimal characteristics and best approximation that other feedforward networks do not have. How to realize the adaptive adjustment of the structure of the RBF neural network while optimizing the parameters of the RBF neural network, improve the performance of the RBF neural network, and enhance its application capabilities, is an urgent problem to be solved in the design and application of the RBF neural network. Aiming at the problems of Particle Swarm Optimization (PSO) algorithm that has premature convergence and easy to fall into local convergence, an Adaptive Particle Swarm Optimization (APSO) algorithm is designed. Using the diversity of particle populations and the flight status information of individual particles, we adaptively adjust particle flight parameters to better prevent particles from falling into local convergence and balance the global and local search capabilities of particles. The experimental results show that the APSO proposed in the article has higher search accuracy than other improved PSOs. By analyzing the characteristics of RBF neural network parameter optimization, PSO is used to optimize RBF neural network parameters. Aiming at the shortcomings of standard PSO algorithms that are easy to fall into local optimality, the main influencing factors of PSO global search and local search are analyzed. Based on particle flight information, an adaptive inertial weight adjustment strategy is proposed, APSO algorithm is designed, and it is used to optimize RBF neural network parameters. The competition of sports performance is essentially a contest of competitive ability. Therefore, good competitive ability is an important guarantee for achieving excellent sports performance. It determines the level of athletes' competitive ability. Only by developing athletes' competitive ability can their sports performance be improved. Competitive ability refers to the ability of athletes to participate in competitions. It is a comprehensive manifestation of the skills, physical stamina, and psychological abilities that should be possessed in competitive competitions. The structure of the following article is as follows: in Section 2, we devote to the discussion of related work; in Section 3, we research on athlete's competitive ability evaluation research method; in Section 4, a radial basis function neural network based on APSO optimization is designed; in Section 5, we devote to APSO-RBF neural network athletes' competitive ability evaluation results and analysis; Section 6 is contributed to the conclusion of the full text.

RETRACTED

## 2. Related Work

Relevant scholars pointed out that, driven by big data, the transplantation of wearable device technology should be actively explored [7–9]. It can actively build an information management platform for athlete training and competition, which is conducive to the big data integration of valuable data information such as functional consumption, technical tracking, and tactical analysis. In the way of mobile data transmission, the coach can realize the visualization of the adjustment of the on-site athletes' functional level and the adjustment of technical and tactics, which can form a complete information of the athletes' training, and competition, which is strongly supported by science and technology [10–12].

Among the many artificial neural networks, RBF neural network has become a research hotspot of Chinese and foreign scholars in recent years due to its bionics background, simple network structure design, and solid mathematical foundation [13–15]. The RBF neural network has only one hidden layer. The hidden layer is composed of nonlinear radial basis functions, but the hidden layer to the output layer is linear. Therefore, optimization algorithms can be used to solve problems such as local minimums. Compared with other neural networks, the main advantage of RBF neural network is that, in addition to its simple structure, it can use nonlinear functions to locally approximate nonlinear input and output mappings. It has a global nonlinear approximation function, because the local adjustment of neurons is faster [16–18]. RBF neural network has been successfully applied to engineering fields such as pattern recognition, image processing, data analysis, nonlinear function approximation, system modeling, information processing, time series analysis, control, and fault diagnosis.

Many early SLFN-type networks used the first randomly selected training data point as the center of the RBF neuron when setting their network parameters and then used singular value decomposition to solve the weight (or height) of the RBF neuron. Relevant scholars use K-means clustering method to determine the center of the radial basis function [19, 20]. This method is widely used in the learning of RBF networks, but this algorithm is sensitive to the initial center of the clustering. Researchers have created a method that uses gradient descent training to select RBF centers [21]. This algorithm is called Generalized Radial Basis Function (GRBF). The Orthogonal Least Squares (OLS) algorithm proposed by related scholars selects the input data that has the greatest impact on the output of the network as the center of the neuron and adds it to the RBF network one by one until the appropriate network is constructed [16]. This method does not have numerical ill-conditioned problems and is simple and efficient, but the selected network structure is not necessarily the simplest. Researchers have also proposed Regularized Orthogonal Least Squares (ROLS) [22]. Combining the OLS method and the regularization method can train an RBF network with simple and generalized network structure and superior performance. Relevant scholars use key vectors instead of cluster centers to construct RBF networks, first use Support Vector Machine (SVM) to calculate support vectors, and use these vectors as the centers of neurons [23]. Experiments show that the RBF network based on support vector has better performance than the usual RBF network.

RETRACTED

At present, more and more RBF neural network algorithms based on a small number of RBF neuron training problems have been proposed [24, 25]. During the training process, there is a period called the “growth cycle.”; In this cycle, a neuron that meets two splitting criteria splits into two new neurons. This learning scheme provides a framework for combining existing supervised and unsupervised training algorithms into growing RBF neural networks. The Growing and Pruning-RBF (GAP-RBF) algorithm evaluates the “meaning” of each neuron based on the average contribution of the neuron to the network output through all input data [26]. After the neuron is evaluated, it may remain in the network or be eliminated. This process can greatly reduce the network size and training time required to solve the problem [27, 28].

## 3. Athlete's Competitive Ability Evaluation Research Method under the Big Data Platform of Competitive Information Management

### 3.1. Athlete's Competitive Information Management Big Data Platform

The application of big data can effectively expand the dimensions of physical data indicators in the selection of youth competitive sports, the dimensions of physical and biochemical data indicators related to techniques and tactics, and the relevant objective data indicators that effectively describe the impact of psychological factors on athletes, which can effectively resolve subjective factors [29]. The problem of lack of objective basis provides more objective guidance for the selection of talents and the whole work of cultivating talents, as well as scientific basis for coaches.

Using modern technology to collect a large amount of data and freeing limited coach resources from the tedious daily technical statistical work has been applied in other competitive events similar to table tennis. Some well-known domestic coaches and research scholars have paid great attention to this. The intelligent motion sensor monitors the movement trajectory of the athlete's swing technology in real time through the 6-axis multidimensional motion sensor and transmits the monitored data to the background simulation device for processing in real time. The software provides real-time radar graphic feedback, and finally all the sports in the training class are visually displayed, and finally a large amount of visualized data is formed. In addition to analyzing the characteristics of athletes' hitting characteristics, offensive strategies, and physical fitness, “USENSE” can also capture and analyze movement characteristics in real time based on the racquet's trajectory, allowing coaches to quickly and comprehensively understand the real-time data of the athlete's overall sports status and also help athletes achieve technical skills. Based on the analysis results, it provides a clearer direction for the formulation of the players' playing style and tactics, thus organically integrating traditional teaching methods and big data analysis methods.  Figure 1 shows the big data platform for athletes' competitive information management.

RETRACTED

### 3.2. AHP

The basic principle of analytic hierarchy process (AHP) is to decompose a relatively complicated problem into multiple single small problems, each small problem has its influence elements, and then these influence elements are classified and grouped according to a certain relationship. It is also a method that can make decisions on some relatively complicated and vague problems, especially for some problems that are difficult to quantitatively analyze. The idea and steps of using the analytic hierarchy process to calculate the weight are shown in Figure 2.

### 3.3. Fuzzy Comprehensive Evaluation Method

The fuzzy comprehensive evaluation method is mainly used to make an overall evaluation of the competitive ability of badminton athletes. Through the conversion of qualitative evaluation into quantitative evaluation, plus its clear and systematic results, a scientific comprehensive evaluation is finally obtained [30]. The research design framework of this study is shown in Figure 3.

## 4. Radial Basis Function Neural Network Design Based on APSO Optimization

### 4.1. RBF Neural Network

RBF neural network is a typical feedforward neural network. The structure of RBF neural network is generally composed of three layers: input layer, hidden layer, and output layer. The input layer directly maps the input vector to the hidden layer as the hidden layer input. From the input layer to the hidden layer is a nonlinear mapping, and from the hidden layer to the output layer is a linear mapping; that is, the output of the network is the linear weighted sum of the output results of the hidden layer.

RETRACTED

The hidden layer performs a nonlinear transformation on the input vector, maps the low-dimensional input vector to the high-dimensional space, and solves the unsolvable problems in the low-dimensional space in the high-dimensional space. The output of the kth neuron in the hidden layer is

(1) $$\begin{array}{c} \phi_{k}\left(x\right)=\sigma_{k}^{2}\cdot \left(e^{u_{k-1}}-x\right). \end{array}$$

Among them, *ϕk* is the output of the kth hidden layer neuron, and *μk* and *σk*, respectively, represent the center and width of the kth hidden layer neuron. During the training process, the center and width will be dynamically adjusted according to the sample. *k* = 1, 2,…, *K*, *K* is the number of neurons in the hidden layer.

The third layer is the output layer, which responds to the output of the hidden layer. The mapping function is a linear function, which is a linear combination of the output results of each hidden layer by connecting the weights. The expression is as follows:

(2) $$\begin{array}{c} y=\underset{K⟶\infty }{\lim}\prod_{k=0}^{K}\phi_{k+1}\cdot w_{k}, \end{array}$$

and among them, *w*_*k*_is the connection weight between the *k*th hidden layer neuron and the output of the network. According to the structure of the RBF neural network, the parameters of the RBF neural network include the center value *μk*, the width *σk*, and the connection weight wk. These three parameters ultimately determine the performance of the neural network. Therefore, how to better optimize the RBF neural network parameters appears especially important.

### 4.2. RBF Neural Network Parameter Optimization

When the structure is determined, the RBF neural network parameters determine its final performance. In the early stage of RBF research, parameter optimization is the focus of RBF neural network research. The study found that when the center and width of the RBF neural network are determined, the network becomes a linear equation set from input to output. At this time, the connection weight of the output layer can be solved by a simple gradient method. The so-called optimization algorithm is actually a search process or rule. It is based on a certain idea and mechanism to obtain an optimized solution that meets the user's requirements through a certain way or rule.

According to the different methods of selecting the RBF function center, the learning of RBF neural network parameters mainly includes gradient and evolutionary algorithms. The development of gradient methods takes a long time and has produced many better algorithms, such as gradient descent, Newton and LM algorithms, and so on. Among them, the error backpropagation (BP) algorithm is the simplest gradient algorithm, and it is also the most popular and widely used algorithm. However, the BP algorithm takes a long time to converge and has poor global search capabilities. Compared with the BP algorithm, the recursive least squares (RLS) algorithm has a faster convergence speed. However, the RLS algorithm involves more complex mathematical operations and more computational space.

RETRACTED

Genetic algorithm mainly includes selection, crossover, mutation, and other processes. The crossover mutation of genetic algorithm makes it have a stronger global search ability, but its complex operation process also makes its initialization parameters more and computational complexity increase. The PSO algorithm does not have the cross-mutation operation of genetic algorithm. In the process of particle search, the search direction is adjusted according to the information transmitted by other particles and the information of the particle itself. This update mode makes the particle swarm structure simple and has fewer operating parameters. Compared with other evolutionary algorithms, PSO has a faster convergence speed. Therefore, it has attracted more and more attention in practical applications and has become a hot research object.

However, evolutionary algorithms have common shortcomings, which may lead to overfitting learning; in particular, when the search space is huge, evolutionary algorithms will produce greater computational complexity. In addition, the analysis of its convergence is still not perfect, and the algorithm convergence cannot always be guaranteed. In the paper, the standard PSO algorithm will be improved and the convergence of the PSO optimized RBF neural network will be analyzed.

### 4.3. APSO Algorithm Construction

PSO algorithm is a random search algorithm based on population, which originated from the study of foraging behavior of bird flocks, by simulating the cooperative behavior during the flight of a flock of birds, designing the mutual cooperation and information sharing mechanism between particles, remembering the historical movement information of themselves and the group, and updating their flight speed and flight position through the sharing of information between themselves and other individuals. In the search process, the particles continuously judge the feasible area and update the current position, so as to better find the best in the complex space. According to this intelligent behavior, the PSO algorithm was proposed and used to solve many optimization problems, and it has been widely used in optimizing neural networks.

RETRACTED

#### 4.3.1. PSO Algorithm

Each particle in the PSO algorithm is regarded as a solution in the D-dimensional feasible solution space, and the particle position can be expressed as

(3) $$\begin{array}{c} L_{i}=\left(L_{i0},L_{i1},L_{i2},...,L_{iD}\right). \end{array}$$

Among them, *D* is the dimension of the search space, *i* = 1, 2,…, *s*, *s* is the number of particles. And the particle velocity can be expressed as

(4) $$\begin{array}{c} X_{i}=\left(x_{i0},x_{i1},x_{i2},...,x_{iD}\right). \end{array}$$

Update the particle individual optimal through the particle fitness value, as shown in the following formula:

(5) $$\begin{array}{c} p_{i}\left(t+1\right)=\left\{\begin{array}{cc} L_{i}\left(t+1\right) & f\left[L_{i}\left(t+1\right)\right]<f\left[p_{i}\left(t\right)\right]\\ p_{i}\left(t-1\right) & f\left[L_{i}\left(t+1\right)\right]\geq f\left[p_{i}\left(t\right)\right] \end{array}\right). \end{array}$$

Among them, the function *f*(*ai*(*t*)) is the fitness function, which is used to express the pros and cons of the solution. In different search periods, the group needs different global search capabilities and local search capabilities, so that particles are not easy to fall into local minima and can find the global optimal solution. In order to better balance the global and local search capabilities of the population, inertial weights are introduced on the basis of the original PSO algorithm. The speed update formula is as follows:

(6) $$\begin{array}{c} x_{id}\left(t+1\right)=wx_{id}\left(t\right)-c_{1}r_{1}\left[p_{id}\left(t\right)-a_{id}\left(t\right)\right]-c_{2}r_{2}\left[g_{d}\left(t\right)-l_{id}\left(t-1\right)\right]. \end{array}$$

Among them, *ω* is the weight of inertia, *c*_1_, *c*_2_ are acceleration constants, usually *c*_1_ = *c*_2_, and generally take a value in [0,2]. *r*_1_ and *r*_2_ are random numbers uniformly distributed in [0, 1].

#### 4.3.2. APSO Algorithm

For the PSO algorithm, diversity plays an important role in improving the effect of evolution. The manifestation of premature convergence of particles is the lack of diversity. The inertia weight plays an important role in adjusting the particle flight. In order to improve the diversity of the algorithm, the inertia weight will be adjusted according to the particle space state. In addition, since the flight of particles is not a simple linear process, this paper proposes a nonlinear adaptive strategy based on group diversity to adjust the inertia weight. The definition of diversity is

(7) $$\begin{array}{c} S\left(t\right)=\frac{f_{\max}\left[l\left(t\right)\right]-f_{\min}\left[l\left(t\right)\right]}{f_{\max}\left[l\left(t\right)\right]+f_{\min}\left[l\left(t\right)\right]}. \end{array}$$

Among them, *f*(*ai*(*t*)) is the fitness value of the *i*-th particle, *i* = 1,2, ..., s, and *f*_min_((*t*)) and *f*max((*t*)) are the minimum and maximum fitness at time *t*, respectively. The diversity *S*(*t*) is used to describe the movement characteristics of particles, represents the degree of aggregation and dispersion of particles, reflects the overall search state of the group, and can reflect the information that the particles fall into the local optimum. We design a nonlinear regression function based on the diversity *S*(*t*) to adjust the inertia weight to make it more in line with the particle flight state. The nonlinear function is as follows:

(8) $$\begin{array}{c} \gamma \left(t\right)={\left[\theta -S\left(t-1\right)\right]}^{-t}. \end{array}$$

Among them, *θ* is the initialization constant, and *θ* ≥ 3. In addition, the spatial state of each particle is different, and the inertia weight needs to be adjusted adaptively according to the state of the particle to guide the flight of each particle. The difference between the particle and the optimal particle can well reflect the current optimal difference of the particle, thereby guiding the flight of the particle. The difference between the particle and the optimal particle is expressed as

(9) $$\begin{array}{c} L_{i}\left(t\right)=\frac{f\left[g\left(t\right)\right]-f\left[l_{i}\left(t\right)\right]}{f\left[g\left(t\right)\right]+f\left[l_{i}\left(t\right)\right]}. \end{array}$$

Among them, *f*(*g*(*t*)) is the global optimal fitness value. Based on the above analysis, the adaptive inertia weighting strategy is defined as

(10) $$\begin{array}{c} w_{i}\left(t\right)=\gamma \left(t-1\right)\cdot \left[L_{i}\left(t-1\right)-\beta \right], \end{array}$$

where *ωi*(*t*) is the inertia weight of the *i*-th particle at time *t* and *β* ≥ 0 is a predefined constant to improve the particle's global search ability.

RETRACTED

In order to further improve the local search ability of the particle in the later stage, a particle velocity range limitation formula is proposed, which makes the particle velocity range gradually shrink as the iteration progresses, thereby enhancing the local search ability:

(11) $$\begin{array}{c} \left\{\begin{array}{c} x_{\min}=\left(N-1\right)\cdot u^{-\text{iter}}\\ x_{\max}=\left(N+1\right)\cdot u^{-\text{iter}} \end{array}\right). \end{array}$$

Among them, *N* is a constant, the value range is [0, 1], the value range of *u* is [1, 1.1], and iter is the number of current iteration steps. By improving the inertia weight adjustment formula and increasing the speed range adjustment formula, the APSO algorithm is proposed, which can better balance the global search ability and local search ability of the PSO algorithm.

### 4.4. APSO-Based RBF Neural Network

In the RBF neural network, the parameters are distributed in the hidden layer and the output layer. The output of the kth neuron in the hidden layer is

(12) $$\begin{array}{c} \phi_{k}\left(x\right)=\sigma_{k}^{2}\cdot e^{\left|u_{k}-x\right|}. \end{array}$$

The network output is

(13) $$\begin{array}{c} y=\underset{K⟶\infty }{\lim}\prod_{k=0}^{K}\phi_{k}\cdot w_{k+1}. \end{array}$$

Therefore, the neural network parameters include the center value *μk*, the width *σk*, and the connection weight *w*_*k*_. The dimension of particle space is

(14) $$\begin{array}{c} D=\left(n+1\right)\cdot \left(K+1\right). \end{array}$$

Among them, *n* is the number of input variables, and *K* is the number of neurons in the hidden layer. In order to use the powerful search capability of the APSO algorithm to minimize the network error function and achieve the network prediction effect, the relative error function (RMSE) between the actual output of the sample and the network output is used as the fitness function of the APSO algorithm. The fitness function formula is as follows:

(15) $$\begin{array}{c} f\left[x_{i}\left(t\right)\right]={\left[\frac{1}{Z}\underset{T⟶\infty }{\lim}\prod_{t=0}^{T}\left|yd\left(t\right)-y\left(t\right)\right|\right]}^{1/2}. \end{array}$$

Among them, yd(*t*) is the actual output, *y*(*t*) is the network output, and *Z* is the number of samples. The detailed process steps of APSO-RBF neural network are shown in Figure 4.

## 5. APSO-RBF Neural Network Athletes' Competitive Ability Evaluation Results and Analysis

### 5.1. APSO-RBF Neural Network Nonlinear Identification Experiment

In this experiment, APSO-RBF neural network is applied to nonlinear system identification. The training input is divided into two parts, half of which are uniformly distributed in [−1, 1], and the other half of the input is determined by the sinusoid function 1.01 × sin(t/45). The test input *u*(*t*) is a piecewise function. This nonlinear system is used to verify the performance of the neural network, 300 sets of training samples and test samples each. In order to verify the performance of the proposed method, APSO-RBF is compared with other RBF neural network structures, as shown in Figure 5.

The results of time series prediction and nonlinear system simulation experiments show that APSO-RBF has a better prediction effect for nonlinear systems; that is, it has higher accuracy. Moreover, the improved APSO has better optimization performance for RBF. Compared with other PSO optimized RBF neural networks, APSO-RBF has the lowest error rate.

RETRACTED

### 5.2. Comparative Analysis of Athletes' Competition Scores

The final form of athletic ability is athletic performance, which is the most intuitive quantitative reflection of athletic ability level. The ultimate goal and task of athletic training is to win ideal athletic performance. The quality of athletic performance is mainly determined by ranking. The ranking is mainly determined by the athletes' scores. According to the characteristics of competitive sports and the rules of international Nanquan routine competition, Nanquan scores are mainly based on the superposition of the three parts of the action quality, the performance level, and the difficulty of the action. Therefore, the sports performance of sports events is mainly determined by three aspects: the quality of the action, the level of practice, and the difficulty of the action. In order to have a clearer understanding of the competitive ability of outstanding athletes, this article conducts a statistical analysis of sports competitions.

#### 5.2.1. Overall Evaluation and Analysis of Project Competition

A total of 100 athletes participated in the sports finals. Since the research object of this article is excellent athletes, the statistics of this article are all above 9.0 points. It can be seen from Figure 6 that the results of APSO-RBF algorithm evaluation are closest to the true value.

#### 5.2.2. Statistical Analysis of Project Action Quality Score

It can be seen from Figure 7 that APSO-RBF has very little difference between the action quality scores of 100 athletes and the real values, which shows the effectiveness of APSO-RBF on the action quality scores of outstanding athletes.

#### 5.2.3. Analysis of Project Performance Level Scores

The scoring situation of the drill level is shown in Figure 8. In terms of exercise level, APSO-RBF still achieved the best evaluation results because its evaluation value is the closest to the real value.

#### 5.2.4. Analysis of the Difficulty Score of the Project Action

It can be seen from Figure 9 that most athletes were evaluated by APSO-RBF score close to 1.65 points on the difficulty of movement, which is generally coincident with the true value. The evaluation value of the other two algorithms is around 1.6.

#### 5.2.5. Index Evaluation of Athletes' Competitive Ability

Competitive ability refers to the ability of athletes to participate in competitions. It is composed of physical stamina, skills, psychology, and intelligence with different manifestations and different functions and is comprehensively manifested in the process of special competitions during competitions. Competitive ability includes physical ability, skills, mental ability, tactical ability, and knowledge ability. Among them, physical ability can be divided into physical form, physical function, and sports quality. Competitive ability is not only a comprehensive manifestation of physical stamina, skills, and mental abilities, but also the expression of artistic value. The momentum and ferocious expressions in the arena can win a decisive victory in competitive competitions under certain circumstances.

RETRACTED

Competitive performance is the most direct manifestation of competitive ability. According to the statistical analysis of sports competition performance, competitive performance is mainly determined by the quality of the exercise, the level of exercise, and the difficulty of the exercise. Among them, the exercise is the main part that determines the competitive performance of outstanding athletes. Secondly, the quality of the action is lower. Therefore, the statistics of the content of the elite athletes' competitive ability indicators must serve the practice level, movement difficulty, and movement quality as the main purpose. To successfully complete each movement difficulty, you must have the physical stamina required to ensure the smooth completion of the movement. The level of practice is not only the expression of movement strength, rhythm, music, etc., but also the embodiment of the athlete's psychological ability and artistic expression, and the quality of the movement. The completion must be based on superb skills. Therefore, according to the characteristics of sports events and sports training theories, we can draw up the primary indicators of outstanding athletes' competitive ability as physical fitness, skills, mental skills, artistic performance, and tactical skills.

According to the characteristics of sports events, each indicator plays a different role in Nanquan's competitive ability system. There are main indicators, secondary indicators, and useless indicators. The importance of the ability is evaluated, the important subabilities are retained, and the unimportant subabilities are eliminated. This article invites 20 experts to use five levels of evaluation and assignment for each indicator based on its important conditions; that is, “very important” is assigned a value of 10, “important” is assigned a value of 7–9, “general” is assigned a value of 4–6, and for “not very important” we assign a value of 1–3 and assign a value of 0 for “not important”. After the expert scores are assigned, the weighted method is used to perform statistical analysis on the obtained data, as shown in Table 1.

It can be seen from Table 1 that the scores of 4 indicators of skill, athletic quality, artistic performance ability, and mental ability are all above 5 points, which are important indicators. The degree of importance is fair, so it is removed. Therefore, the main constituent elements of competitive ability are skills, athletic qualities, artistic performance ability, and psychological ability.

RETRACTED

The four elements of athletes' competitive ability are also in line with the development law of competitive sports, because according to the performance evaluation criteria of competitive Nanquan, the final performance of competitive Nanquan is determined by the quality of the action, the level of exercise, and the difficulty of the action. This kind of movement and the performance of superb skill level must have good athletic quality and good mental ability as well as good artistic expression. Good athletic quality provides a source of motivation for the completion of Nanquan skills, and good psychological quality provides a stable environment for the completion of skills. Good artistic expression makes the skill movements more perfect.

## 6. Conclusion

Under the influence of the wide application of big data, we make full use of its advanced information technology and other successful experience in big data in competitive sports, effectively combine big data with athletes' competitive work, and strive to reduce blindness and blind obedience in the competitive stage. The dynamic optimization of the RBF neural network structure is an effective method to ensure that the RBF neural network always works in a suitable structure state. In order to obtain an effective method for the dynamic adjustment of the RBF neural network structure, the RBF structure is adjusted according to the change of the task. On the basis of in-depth analysis of the existing research results, an APSO-based RBF neural network structure optimization design method is proposed. This solves the problem that the RBF neural network structure does not match the actual task and realizes the simultaneous adjustment of the RBF neural network structure and parameters, thereby improving the performance of the RBF neural network. The results of this article show that competitive strength is the core of athletes' competitive ability, and ability to play is the key to athletes' competitive ability. Competitive strength is the main factor, which directly determines the level and stability of the athlete's competitive level. Ability to play is a secondary factor, which is related to whether the athlete can smoothly or even supernormally transform competitive strength into sports performance. By weighting the second-level indicators, the weights of the second-level indicators of athletes' competitive ability are in order of skill, athletic quality, psychological ability, and artistic expression. Skills are the main factors that determine the level of competitive ability. Sports quality and psychological ability are important guarantees for supporting the normal performance of skills. Artistic expressiveness is a supplementary factor for competitive ability. The various elements cooperate with each other and interact with each other. The indicators do not exist alone but cooperate with each other to support the formation of the entire athletic ability system. In the content of the competitive ability index of excellent athletes, technical ability is the core, and sports quality, psychological ability, and artistic performance ability ultimately exist to serve the improvement of technical ability.

RETRACTED

## Figures and Tables

**Figure 1:** Athlete's competitive information management big data platform.

**Figure 2:** The construction process of the evaluation index system of athletes' competitive ability.

**Figure 3:** The research and design framework of this paper.

**Figure 4:** Adaptive particle swarm optimization algorithm.

**Figure 5:** PSO algorithm optimization RBF effect comparison.

**Figure 6:** Overall performance evaluation.

**Figure 7:** Statistics of action quality scores.

**Figure 8:** Statistics of practice level scores.

**Figure 9:** Evaluation of action difficulty score.

**Table 1:** Assignment of the importance of the first-level indicators of competitive ability.

Index	Skills	Athletic fitness	Artistic expression ability	Mental ability	Body function	Body shape	Tactical ability
Assigned total score	221	218	212	209	122	118	107
Assigned average score	9.3	9.2	9	8.7	4.8	4.6	4.3
Ranking	1	2	3	4	5	6	7

## Data Availability

The data used to support the findings of this study are available from the corresponding author upon request.
